# Somatotopy in the Medullary Dorsal Horn As a Basis for Orofacial Reflex Behavior

**DOI:** 10.3389/fneur.2017.00522

**Published:** 2017-10-10

**Authors:** W. Michael Panneton, BingBing Pan, Qi Gan

**Affiliations:** ^1^Department of Anesthesiology, School of Medicine, Washington University in St. Louis, St. Louis, MO, United States; ^2^Department of Pharmacological and Physiological Science, School of Medicine, Saint Louis University, St. Louis, MO, United States; ^3^Department of Anesthesiology, Hunan Provincial People’s Hospital, Changsha, China

**Keywords:** trigeminal, onion skin theory, lamina V, facial motor nucleus, trigeminocervical complex

## Abstract

The somatotopy of the trigeminocervical complex of the rat was defined as a basis for describing circuitry for reflex behaviors directed through the facial motor nucleus. Thus, transganglionic transport of horseradish peroxidase conjugates applied to individual nerves/peripheral receptive fields showed that nerves innervating oropharyngeal structures projected most rostrally, followed by nerves innervating snout, periocular, and then periauricular receptive fields most caudally. Nerves innervating mucosae or glabrous receptive fields terminated densely in laminae I, II, and V of the trigeminocervical complex, while those innervating hairy skin terminated in laminae I–V. Projections to lamina II exhibited the most focused somatotopy when individual cases were compared. Retrograde transport of FluoroGold (FG) deposited into the facial motor nucleus resulted in labeled neurons almost solely in lamina V of the trigeminocervical complex. The distribution of these labeled neurons paralleled the somatotopy of primary afferent fibers, e.g., those labeled after FG injections into a functional group of motoneurons innervating lip musculature were found most rostrally while those labeled after injections into motoneurons innervating snout, periocular and preauricular muscles, respectively, were found at progressively more caudal levels. Anterograde transport of injections of biotinylated dextran amine into lamina V at different rostrocaudal levels of the trigeminocervical complex confirmed the notion that the somatotopy of orofacial sensory fields parallels the musculotopy of facial motor neurons. These data suggest that neurons in lamina V are important interneurons in a simple orofacial reflex circuit consisting of a sensory neuron, interneuron and motor neuron. Moreover, the somatotopy of primary afferent fibers from the head and neck confirms the “onion skin hypothesis” and suggests rostral cervical dermatomes blend seamlessly with “cranial dermatomes.” The transition area between subnucleus interpolaris and subnucleus caudalis is addressed while the paratrigeminal nucleus is discussed as an interface between the somatic and visceral nervous systems.

## Introduction

Much behavior is reflex in nature and serves basic vegetative functions that are usually less complex and more uniform across species. Most reflex circuits consist of a sensory neuron, a variable number of interneurons, and a motor neuron. For example, blinking, chewing, facial expression, even diving behavior, etc., are accomplished mostly without conscious thought, driven by central circuits (or pattern generators) coordinating sensory inputs to motor outputs. Neural circuits located within the brainstem and spinal cord provide the substrate for simple behaviors as well as more complicated circuits influencing orofacial behaviors (1). Our laboratory has sought mostly neuroanatomical evidence for brainstem circuits driving behaviors. We have focused on a somatoautonomic reflex in the past, the mammalian diving response, and established a foundation of neural areas purportedly important for the cardiorespiratory sequelae induced by underwater submersion (2–5), but the finer details of this circuitry are still unknown. We also previously speculated on circuitry involved in the blink reflex (6, 7). The present review examines reflex circuits linked to head and neck sensory nerves/receptors that transmit *via* the trigeminocervical complex to the facial motor nucleus.

There are two commonly taught schemas of innervation of the spinal somatosensory system. One shows the body and limbs innervated by individual cutaneous nerves, circumscribing the average extent of the cutaneous receptive fields of these nerves on the body’s surface. Another pattern illustrates the innervation of individual spinal nerves into dermatomes. The trigeminal homolog of the spinal distribution scheme is the tripartite innervation distribution of the ophthalmic (V1), maxillary (V2), and mandibular (V3) nerves. However, contrasting with the more contiguous dermatomal lines of the upper neck, these large nerves encompass peripheral receptive areas from rostral cervical dermatomes to inside the mouth. Déjerine (8), a French neurologist, proposed an “onion skin theory” of innervation of the face. He described sensory loss in humans starting from the mouth and nose and extending concentrically outward after vascular lesions of the caudal spinal trigeminal nucleus. Graphic representation of the layers of onion skin on the face, ending rostrally as a circling around the nares and mouth, mimics the dermatome pattern of the body—creating “cranial dermatomes.” Such mimicry could only be considered hypothetical, however, since head regions are not innervated by spinal nerves and thus cannot be considered dermatomes *per se*.

We also must remind that somatosensation in the head integrates several unique receptive fields (e.g., teeth, cornea, mucosae of the mouth, nose, and sinuses) which are not found in the lower body. These are innervated overwhelmingly by small diameter fibers and with few, if any, peripheral receptors associated with hairs. Nevertheless, all of these select receptive fields are represented centrally in the rostral medullary dorsal horn (MDH); one would expect the architecture of the central nervous system to adapt to these unique receptive fields.

The known somatotopy of the MDH consists of representations from the mandibular nerve (V3) most dorsally and rostrally, that from V1 most ventrally and caudally, and that from the V2 at intermediate positions. The representation from nerves emanating from cervical dorsal primary rami, carrying sensory fibers innervating dorsal parts of the neck, are continuous rostrally with the V1 nerve of the trigeminal; both project centrally to ventral parts of the spinal and MDHs, respectively. Nerves emanating from ventral primary rami and innervating the ventral neck continue rostrally into dorsomedial parts of the MDH, overlapping with the V3 trigeminal nerve. The continuity of the spinal and MDHs is collectively termed the *trigeminocervical complex*, a term used throughout this treatise. We hypothesize that the somatotopy of the trigeminocervical complex of the rodent mimics that first proposed in humans (8) and suggest his “onion skin” theory of innervation of the head and neck in humans is transferred phylogenetically forward along mammalian lines. Nevertheless, few studies have attempted to link trigeminocervical somatotopy to brainstem reflex circuits.

The facial motor nucleus is a unique collection of motor neurons located near the pontomedullary junction. Almost all constituent facial motor nucleus neurons are alpha motor neurons, with few gamma motoneurons (facial muscles carry relatively uniform loads thus minimizing muscle spindles) and few interneurons. Facial motoneurons often cluster, but both the number of clusters and their nomenclature differ by species and investigator, and reports are somewhat inconsistent in describing subgroups. Nevertheless, motoneurons comprising the facial motor nucleus in the brainstem are arranged topographically in all studied species (9, 10). Motoneurons innervating facial muscles surrounding the eye are dorsolateral, those to pinna muscles are dorsomedial, to the upper lip and whiskers are ventrolateral, and to the lower lip and neck ventromedial. These motoneurons innervate the striated facial musculature required for blinking, pinnae movements, vibrissae whisking, and eating, respectively. We hypothesize the somatotopy in the facial motor nucleus is coordinated with that in the sensory representation in the trigeminocervical complex.

Neuroanatomical experiments were performed utilizing conventional tract-tracing methodologies. The transganglionic transport of a cocktail of horseradish peroxidase (HRP) conjugates, specifically HRP bound with wheat germ agglutinin (WGA-HRP) and HRP bound to cholera toxin (BHRP), was utilized for transport of the tracers centrally after its injection into selected peripheral nerves or receptive fields, with our emphasis placed on projections into the MDH. Retrograde transport of another tracer, FluoroGold (FG), was utilized after its iontophoretic injection into different functional areas of the facial motor nucleus (FN) to determine the location of MDH projection neurons. The anterograde transport of biotinylated dextran amine (BDA) after its iontophoretic injection into different levels of the trigeminocervical complex substantiated the retrograde results, showing a topography. Explanations of these techniques, as well as their pitfalls, are detailed in past publications (7, 11, 12).

Our conventional neuroanatomical data show that primary afferent fibers terminating in the trigeminocervical complex of the rat conform to the “onion skin” hypothesis originally proposed in humans (8). We also show that trigeminal-facial projection neurons, almost all of which are in lamina V of the trigeminocervical complex, faithfully connect homologous parts of body images outlined for both the trigeminocervical complex and facial motor nucleus. This arrangement promotes simple, organized, and mostly automatic circuits that probably form the basis for orofacial reflex behavior.

## Transganglionic Experiments

Transganglionic tracer experiments showed robust labeling in the medullary and spinal dorsal horns after transport in sensory fibers of a particular nerve. Detailed analyses of projections from sensory inputs from the glossopharyngeal, anterior ethmoidal, infraorbital, supraorbital nerves, or from the conjunctiva and cornea have been done previously and will not be repeated herein (7, 12, 13). Nevertheless, the projections of these nerves are included in Figure 1 so that the progression of label from nerves innervating different orofacial areas can be qualitatively evaluated and reinforce our conclusions of a logical order to the somatotopy of orofacial representation in the trigeminocervical complex. The mixture of two different conjugates of HRP, WGA-HRP labeling small fibers preferentially and BHRP labeling large fibers preferentially, differed from most previous studies and greatly enhanced the interpretability of the data.

**Figure 1:** Line drawings showing the distribution of reaction product in the trigeminocervical complex after transganglionic transport of an horseradish peroxidase (HRP) cocktail of tracers injected into individual nerves/receptive fields. Drawings are arranged with rostral sections placed near the top of the figure while more caudal sections are shown near the bottom. Note that nerves/receptive areas innervating glabrous surfaces, e.g., IX–X, lingual, anterior ethmoidal, conjunctiva and cornea, project mostly to laminae I, II, and V, while those innervating hairy skin, e.g., inferior alveolar, infraorbital, supraorbital, and cervical, densely project to all laminae. Bands of color have been arbitrarily superimposed over these drawings; compare these to similarly colored bands on Figure 5. While all nerves have appropriate central projections to areas of the trigeminocervical complex known to represent V1, V2, and V3 divisions of the trigeminal nerve, the rostrocaudal distribution of the reaction product from different nerves imply the existence of “cranial dermatomes.” Note the progression of reaction product in the trigeminocervical complex from nerves innervating oral and perioral areas rostrally (upper left corner of figure with red hue) toward those innervating the snout (in the middle shaded green), periocular areas (in the middle shaded blue), to finally cervical dermatomes (in the lower right corner shaded orange). The central representation of the cornea, however, defies the maps order and is drawn as the last column. Numbers adjacent to line drawings represent mm caudal to the obex.

Discrete areas of the trigeminocervical complex relative to either the dorsoventral or rostrocaudal axes contained localized patches of tracer for each nerve (Figure 1). Transported label was robust in laminae I–V of the trigeminocervical complex from the infraorbital, supraorbital, inferior alveolar (also a conduit for the mental nerve), and cervical nerves; all these nerves densely innervate hairs. In contrast, more restricted dense labeling occurred in laminae I, II, and V, but just sparse label in laminae III and IV, for projections arising from the glossopharyngeal/vagus, lingual, anterior ethmoidal nerves, the cornea and conjunctiva. The receptive fields of these latter nerves contain few, if any, hairs. Reaction product in lamina II was exceptionally intense in all the cases, especially in its inner sublamina from nerves innervating hairs and teeth.

The rostrocaudal distribution of reaction product was consistently not uniform across laminae. Labeling in lamina I of the MDH extended broadly around its curvature and rostrocaudally in both laminae I and V for all studied nerves, suggesting considerable overlap and a blurred somatotopy in these laminae (6, 7, 11–13). There were more restricted projections into laminae III and IV in the rostrocaudal distribution, suggesting possibly more focused somatotopy in these layers. However, lamina II contained the most confined projections with dense reaction product in all cases. Generally, there was minimal overlap from different nerves in lamina II relative to the other laminae. For example, there was minimal overlap in lamina II in the projections at level—0.5–0.6 mm caudal to obex (Figure 1; horizontal row in red zone) and levels—3.0–3.5 mm (Figure 1; middle horizontal row in blue zone).

Label from some nerves indicated projections to areas beyond the ipsilateral trigeminocervical complex. Nerves with cutaneous receptive fields located on the midline showed projections to homologous areas of the contralateral dorsal horn (14–17). Fibers crossed the midline in the dorsal commissure dorsal to the central canal and entered the contralateral dorsal horn (Figure 2A; arrows). Also, injections into the lingual nerve yielded reaction product in the nearby reticular formation extending toward the ipsilateral ventrolateral nucleus of the solitary tract (Figures 1 and 2B–D, arrows). Injections of the glossopharyngeal/vagus and lingual nerves also induced intense labeling in the paratrigeminal nucleus (Figures 1 and 2B,E). This reaction product also continued into the reticular formation (Figures 2B–D) toward the ventrolateral subnucleus of the solitary tract. Injections of the IX/X nerve lead to a line of intense label along the curvature of the rostral MDH at levels of the obex, presumably in lamina I (Figure 2E, arrows). While there was little reaction product in the MDH after IX/X nerve injections beyond the first millimeter caudal to the obex (Figure 1), intense reaction product in the cervical dorsal horn appeared more caudally, possibly representing the innervation of the pinna by these nerves (Figure 2F). Robust reaction product in the cervical dorsal horn covered all laminae in its ventrolateral parts after injections of the greater occipital nerve (Figure 2G).

**Figure 2:** Darkfield photomicrographs illustrating selected projections after transganglionic transport of a horseradish peroxidase (HRP) cocktail injected into different nerves of the head and neck. Injections of cutaneous nerves with receptive fields along the midline, including the supraorbital and mental (the terminal branch of the inferior alveolar n.) nerves, resulted in reaction product in homologous areas of the contralateral trigeminocervical complex. The route for crossing fibers and their contralateral destination for the mental nerve (inferior alveolar n.) are shown **(A)**. Injections of the lingual nerve resulted in reaction product in the dorsolateral reticular formation, encroaching on the ventrolateral subnucleus of the nucleus of the solitary tract [**(B–D)**; arrows] as well as dense label in laminae I and II of the ipsilateral medullary dorsal horn (MDH) **(D)**. Panels **(B,E)** illustrate the dense reaction product in the paratrigeminal nucleus (Pa5) after injections of the lingual and IX/X nerves. Reaction product is seen in laminae I and II, the nucleus of the solitary tract (NTS), as well as intense label in the presumptive lamina I of the rostral MDH [**(E)**; arrows] after injection of IX/X nerves. It is well known that the glossopharyngeal and vagus nerves have receptive fields on the pinna; **(F)** shows reaction product in the rostral cervical dorsal horn is seen after injection of the IX/X nerves, presumably marking the central representation of the auricle. White arrow in **(F)** points to caudal extension of the solitary tract. Reaction product after transganglionic transport of the HRP cocktail in the greater occipital nerve is seen in all laminae of the ventrolateral cervical dorsal horn **(G)** as well as the central cervical nucleus [**(G)**; arrow].

## Tract Tracing Experiments

In four cases, injections of FG into the facial motor nucleus involved either intermediate (Figure 3A), dorsolateral (Figure 3C), ventrolateral (Figure 3E), or medial (Figure 3G) regions, respectively. Facial motoneurons in different nuclear locations preferentially innervate different target muscles. Intermediate parts innervate lip muscles, those dorsolateral innervate muscles surrounding the eye, ventrolateral motoneurons innervate musculature of the vibrissae and nares, and medial parts innervate pinna and platysma muscles. Interneurons in lamina V of the trigeminocervical complex almost exclusively received retrograde transport of FG after the facial motor nucleus injections (Figures 3B,D,F,H). Moreover, the distribution of the retrograde labeling was not uniform either rostrocaudally or dorsoventrally, despite injections overlapping the functional delineations in the facial nucleus. Thus, trigeminocervical neurons retrogradely labeled after an intermediate facial nucleus injection generally were in the center of lamina V in its rostral half (Figures 3I–L; red squares), those from dorsolateral injections were ventrally located in the rostral third of the MDH (Figures 3I–K; green triangles), those from ventrolateral injections were in its rostral half (Figures 3I–L; blue diamonds), while those from medial injections were mostly in its caudal half (Figures 3L–O; orange circles), but with a few in dorsal rostral parts (Figures 3I,J).

**Figure 3:** Bright field photomicrographs showing FluoroGold injections into intermediate **(A)**, dorsolateral **(C)**, ventrolateral **(E)**, and medial **(G)** parts of the facial motor nucleus and its subsequent retrograde transport into the trigeminocervical complex [**(B)** pairs with **(A)**, **(D)** with **(C)**, **(F)** with **(E)**, and **(H)** with **(G)**]. Note that almost all retrograde labeling in the medullary dorsal horn (MDH) from these cases was found in lamina V [arrows **(B,D,F,H)**]. **(I–O)** are composite line drawings showing the differential distribution of retrograde labeling in lamina V after injections of intermediate (red squares), dorsolateral (green triangles), ventrolateral (blue diamonds) and medial (orange circles) parts of the facial motor nucleus. These areas represent functional groups of motoneurons innervating lip musculature, periocular muscles, snout muscles, and periauricular muscles, respectively. Note that neurons retrogradely labeled after intermediate facial injections generally are found centered in lamina V in the rostral half of the MDH, those from dorsolateral injections are found ventrally in the rostral third of the MDH, those from ventrolateral injections are centered in its rostral half, while those from medial injections are mostly in the caudal half of the trigeminocervical complex, but with a few in dorsal rostral parts. Numbers in **(I–O)** indicate millimeters caudal to the obex. We propose that such retrogradely labeled neurons are important interneurons in simple disynaptic reflex circuits.

Injections of BDA that involved lamina V of trigeminocervical complex at different rostrocaudal levels (Figure 4) produced a topographic pattern of labeling in the facial motor nucleus (Figure 4A). An injection in the rostral-dorsal MDH, where sensory fibers from intraoral receptive fields terminate (Figure 4C; red arrow), resulted in anterograde transport of BDA to intermediate parts of the facial nucleus (Figure 4B; red arrows), where motoneurons innervating lip musculature reside. This injection mainly affected laminae III–IV but also neighboring lamina V. An injection into the ventrolateral part of the rostral MDH (Figure 4E; blue arrow), where sensory fibers from the cornea and anterior ethmoidal nerve project, labeled dorsolateral areas of the facial nucleus (Figure 4D; green arrows), which includes motoneurons innervating the orbicularis oculi muscle. An injection into lamina V of the middle third of the MDH, which receives sensory fibers innervating the snout, selectively labeled ventrolateral parts of the facial motor nucleus (Figure 4F; blue arrows) containing motoneurons innervating vibrissae. Although the injections in Figures 4E,G appear quite large, a feature common to all injections centered in lamina V was uptake and spread of the BDA into the large dendritic arbors of lamina V neurons. An injection into lamina V of the C3–4 level of the rostral spinal cord (Figure 4I; orange arrow), close to where sensory fibers innervating periauricular areas project, produced sparse label in the medial facial nucleus (Figure 4H; orange arrows), containing motoneurons that innervate pinna muscles.

**Figure 4:** Line drawings and photomicrographs illustrating the anterograde transport of biotinylated dextran amine (BDA) into the facial motor nucleus after injections into deep lamina of different rostrocaudal levels of the trigeminocervical complex. Transported label to intermediate parts of the facial nucleus is seen in **(B)** (red arrows) after an injection centered in laminae III–IV of the rostral medullary dorsal horn (MDH) [**(C)**; red arrow]. Similarly, an injection centered in lamina V of the ventrolateral parts of the rostral MDH [**(E)**; green arrow] resulted in transported label to dorsolateral parts of the FN [**(D)**; green arrows] while an injection more caudally in lamina V [**(G)**; blue arrow] labeled ventrolateral parts of the FN [**(F)**; blue arrows]. We suspect appearance of the large size of these injections is due to robust filling of lamina V neurons with dendrites extending to more superficial laminae. Finally, an injection of BDA into lamina V of the C4 level of the spinal dorsal horn [**(I)**; orange arrow] resulted in label in the medial facial nucleus [**(H)**; orange arrows]. These results are summarized in **(A)**; color coding of labeled fibers match those imposed on the different injections at different rostrocaudal levels of the trigeminocervical complex seen in **(B–I)**. When these data are combined with the somatotopy of primary afferent fibers (Figure 1) and retrograde labeling after injections of the FN (Figure 3), a pattern is seen such that homologous body parts represented by sensory systems and motor neurons are tightly coordinated. This synchrony promotes the notion of appropriate simple reflex circuits existing between the somatosensory system and striated motor neurons.

The centripetal transport of markers from nerves innervating oral and facial areas support the hypothesis that a somatotopic scheme exists for linkages in the CNS associated with the representations of all body parts. These cases were all done in rats, with body sizes all within a narrow range, with a similar cocktail of HRP conjugates, and with similar time for transport of the markers. Our transganglionic data support the notion of a progressive continuation of cervical dermatomes into the facial representation, creating perhaps the moniker “cranial dermatomes” in the trigeminocervical complex. These data indicate, and perhaps prove, the “onion skin” hypothesis (8) inspired from observations of facial sensory loss (especially pain and temperature) after vascular stokes of the lateral medulla. Central injections of anterogradely and retrogradely transported markers into either the trigeminocervical complex or discrete functional areas of the facial motor nucleus, respectively, confirm an “onion skin” body representation in the trigeminocervical complex. More importantly, however, these data showed that most trigemino-facial projections arise from neurons in lamina V, thus providing a source for a simple disynaptic reflex circuitry in numerous orofacial reflexes.

Prior discussions assessed the currently utilized transganglionic transport techniques (11–13). The use of both WGA-HRP and BHRP greatly enhanced the findings and interpretations. Consequently, transport of these conjugates was to all laminae and reaction product was generally dense, differing from other reports solely using either WGA-HRP, where reaction product was mostly in laminae I, II, and V, or laminae I, III–V when using BHRP or free HRP.

The presented evidence of a precise somatotopy within the trigeminocervical complex supports the conclusion that the central representation of orofacial receptive fields critically calibrates and directs somatomotor reflex pathways. However, the cytoarchitecture of the rostral MDH, including its transition into the subnucleus interpolaris, can be confusing. The following discussion of the organization of the trigeminocervical system might clarify several issues.

## Anatomy of the Rostral MDH

The paratrigeminal nucleus (Pa5) consists of islands of neuropil in the dorsolateral part of the spinal trigeminal tract near levels of the obex (18). Pa5 receives numerous inputs from several primary afferent nerves. Examples include the IX–X and lingual nerves (Figure 1), the superior laryngeal nerve and receptive areas surrounding the fauces (13, 16, 19–26), and the sensory inputs from the muscles of mastication (27, 28) and molar teeth (26, 29). These studies on projections from primary afferent fibers and other studies (30–32) suggest Pa5 may have a role in ingestion. Others, however, showed that cardiorespiratory activity influences Pa5 (30, 33). Whether Pa5 is a separable entity or a dissociated component of another nucleus is unknown, but its translucent appearance resembles that of the substantia gelatinosa of the MDH (laminae I and II) as well as the gelatinous nucleus tractus solitarii. Consequently, it is of interest that both Pa5 and laminae I and II demonstrate acid phosphatase activity (19, 34, 35), contain similar peptides and amines (36, 37) and send projections into the nucleus tractus solitarii (36, 38). Acid phosphatase activity is also prominent in the caudal nucleus tractus solitarii (39). Collectively, these findings support an earlier suggestion (6, 28) that Pa5 in the dorsal spinal trigeminal tract near obex levels is a probable rostral migration of laminae I and II into the spinal trigeminal tract. The connections of Pa5 also provide support for the hypothesis of a centrally represented unified image of the body. Thus, Pa5 is an interface between the central somatosensory system (represented by the MDH) and the visceral nervous system (represented by the nucleus tractus solitarii). The junction of these two systems peripherally occurs near the oro- and laryngopharynx. Indeed, ours and others data (22, 40) show dense projections from the lingual and glossopharyngeal/vagus nerves spanning the paratrigeminal nucleus into the nucleus tractus solitarii.

The transition between the MDH and the subnucleus interpolaris of the spinal trigeminal nucleus is anatomically complex as are divergent views outlining its organization (41–43). Our view considers the transition from its dorsomedial and ventrolateral aspects. The most rostral pole of the MDH, especially its dorsomedial parts, receives dense primary afferent connections from the IX–X, lingual, and inferior alveolar nerves (Figure 1), especially those from intraoral and associated structures (*vide supra*). We previously noted that sensory fibers innervating mucosae of the head and neck selectively project to laminae I, II, and V of the MDH, sparing laminae III–IV. Since hairs are not found in the mouth and pharynx, sensory fibers innervating them are absent. We suggest that this induces a commensurate depletion of neurons in laminae III–IV centrally, in contrast to the abundance of sensory fibers innervating hairs terminating in the caudal MDH and spinal dorsal horns. Thus, the rostral pole of the MDH appears without strong lamination, and indeed has long been termed *alaminar*, compared to the caudal MDH where cutaneous receptive fields from hairy skin dominate.

The ventrolateral portion of this transition zone is marked by the caudal pole of subnucleus interpolaris, which wedges between the spinal trigeminal tract superficially and the deeper MDH dorsally and medially. The superficial location of lamina II seen in the caudal MDH is thereby displaced medially and the shifted deeper position of lamina II has been called the *displaced substantia gelatinosa*. The displaced substantia gelatinosa is best seen with immunohistochemical studies showing dense label in laminae I and II [for example, see Yoshida et al. (44)]. The present study (Figure 1) and others (12, 13, 45) show this displaced substantia gelatinosa marks the central representation of the anterior ethmoidal nerve, a nerve that innervates the nasal mucosa in part. The representation of the cornea (6, 7) is also nearby (Figure 1). Between these dorsomedial and ventrolateral parts of the transition area is a somewhat laminated portion of the rostral MDH, filled mostly by a representation of the infraorbital nerve (Figure 1), which includes many hairs in its peripheral receptive fields. This conceptualization of the transition between the MDH and subnucleus interpolaris seems plausible to us, especially considering the numerous peripheral receptive fields innervating the hairless mucosae and cornea represented in this transition zone.

## Somatotopy of the MDH

Somatotopy is ubiquitous in the central nervous system but whether it is a product of perception, an epiphenomenon, or musculotopy, its functional significance is unknown (46). If one believes all parts of the body are represented in the central nervous system in a logical manner (e.g., the basis of homunculi superimposed on cortical gyri), one might also suspect that primary afferent fibers innervating discreet regions of the body follow a similar pattern in the dorsal horns. A perspective on somatotopy development is eloquently introduced by Erzurumlu et al. (47), where they summarize embryonic markers directing formation of the somatic representation of whiskers of the rat in the principal trigeminal nucleus, thalamus and cerebral cortex. Unfortunately, they note that nothing is known about the development of somatotopy in the spinal trigeminal nucleus. Nevertheless, it is likely a similar somatotopy exists in the medullary and spinal dorsal horns.

The pioneering degeneration studies of Kerr (48) and several transganglionic transport studies (49–51) unfortunately obfuscated orofacial fibers *descending* in the spinal trigeminal tract with those *ascending* from cervical spinal nerves in the MDH. The problem arose when all these authors chose to ablate/inject dorsal root ganglia rather than individual nerves with discrete peripheral receptive fields. Dorsal root ganglia contain neurons that project peripherally *via* either dorsal or ventral primary rami; Grant (52) showed that dorsal primary rami innervate the most ventrolateral part of the dorsal horn while ventral primary rami innervate dorsomedial parts of the dorsal horn, respectively. Ablation/injection of a whole dorsal root ganglion thus labels both areas of the dorsal horn, confounding statements on trigeminocervical somatotopy. We injected herein a nerve derived from a dorsal primary ramus, and as expected, show dense terminal label in ventrolateral parts of the trigeminocervical complex (Figure 1). Its central terminal fields abut those of the supraorbital nerve, innervating part of our most caudal “cranial dermatome.” We would expect injecting transverse cervical nerves from ventral primary rami innervating the ventral neck therefore would label dorsomedial areas of the trigeminocervical complex and adjoin the central termination of the mental nerve. Nevertheless, similar to our contention for contralateral projections of nerves innervating midline skin (16), a fusion of somatotopy must occur—be it either the right and left sides of the body (Figure 2A) or its dorsal and ventral surfaces. We believe the sparse label in dorsomedial parts of the trigeminocervical complex after injection of the greater occipital nerve (Figure 1, cervical nerve, −2.4 to −3.2) fulfills this fusion of dorsal and ventral body parts on the same side. Again, similar to the homunculus drawn for the cerebral cortex, we believe the whole body is appropriately represented in the dorsal horns.

Thus, our conceived map has the larynx, pharynx, tongue, and oral mucosa represented in the most rostral dorsomedial part of the MDH, including the paratrigeminal nucleus, followed by the snout, periorbital areas then preauricular zones more caudally (Figures 1 and 5). This view is supported by dense reaction product seen in superficial laminae in the first millimeter caudal to the obex after injections of the glossopharyngeal/vagus nerve, and then almost no label (except for lamina I) for at least 5 mm, before a large multilaminar aggregation of reaction product appeared (Figure 2G). We suspect the latter reaction product represents the auricle, innervated by multiple cranial nerves including the glossopharyngeal and vagus, confirming other data (53, 54). Two large nerves, the infraorbital and inferior alveolar, innervate extensive peripheral receptive fields and accordingly span multiple bands of our construed “cranial dermatomes.” The inferior alveolar nerve, innervating mandibular teeth, gingiva over the mandible, as well as skin covering the chin *via* its mental branch, was marked by dense reaction product in the trigeminocervical complex, especially in inner lamina II. The latter reaction product aligns well with data on individual mandibular teeth (27, 55–58), which show dense reaction product in inner lamina II.

The central representation of the cornea, which we believe is dissociated from that of the conjunctiva (6, 7), does not fit in our somatotopic map, however. Similar views have been discussed previously (6, 59). We show most corneal primary afferent fibers project to lamina I (Figure 1), with but little input to lamina II (7), supporting notions that corneal stimulation induces only the sensation of pain. The development of the eye is complex (60) and the corneal epithelium constantly is renewed from stem cells located near the limbus (61), perhaps retarding a formal representation in lamina II, the basis of our somatotopic map. Moreover, the corneal innervation develops only from neurons of neural crest origin, versus other facial cutaneous innervation mostly from placodal origin (62), and perhaps this skews the somatotopy.

The “onion skin” theory of facial innervation has been supported in humans after trigeminal tractotomy (63) and experimentally in several species (6, 26, 34, 35, 64–66). We have discussed this theory in terms of “cranial dermatomes” in continuity with cervical spinal dermatomes, using the term trigeminocervical complex to encompass this merger. However, some (41, 43) debunk this notion based on data from neurons responsive to stimulation of the cornea, temporomandibular joint or masseter muscle. They propose a unique area in the Vi/Vc transition zone, stating the trigeminal system includes areas important for pain processing and autonomic function different from that seen in the rest of the body.

## Trigeminofacial Projections: A Substrate for Orofacial Reflex Behaviors

A reflex by definition is “an involuntary reaction in response to a stimulus applied to the periphery and transmitted to the nervous centers in the brain or spinal cord” (Stedman’s Medical Dictionary). We believe our data promote rather simple circuits that many orofacial reflexes utilize during normal behavior. Thus, injections of FG into functionally discrete regions of the facial motor nucleus induced retrogradely labeling *mostly in lamina V* of the trigeminocervical complex (Figure 3). Such labeling was organized somatotopically similar to that of primary afferent projections but with the caveat that the body image is blurred in lamina V. Thus, most retrogradely neurons labeled after medial facial injections, where motoneurons innervating auricular and platysma muscles occur, were found most caudally. Those retrogradely labeled after ventrolateral facial injections, where motoneurons innervating vibrissae and nares are located, as well as after injections into intermediate facial injections, containing motoneurons innervating the lips, in rostral-middle regions of the trigeminocervical complex. After injections of FG into dorsolateral facial areas, which contain motoneurons projecting to the orbicularis oculi muscle, most retrogradely labeled neurons were found in ventrolateral portions of the rostral trigeminocervical complex (Figures 3I–K) and others were noted more caudally (Figures 3M,N). These areas overlap the central projections of the cornea and conjunctiva, respectively (7). Moreover, injections of BDA into different rostrocaudal levels of the trigeminocervical complex including lamina V neurons showed somatotopically appropriate anterograde projections to the different functional subdivisions of the facial motor nucleus.

This promotes the large multipolar neurons in lamina V as important for trigemino-facial reflex behaviors, as noted previously (67, 68). Indeed, the Vi/Vc area, near to where we show projecting sensory fibers from the cornea, has been shown electrophysiologically to project to dorsolateral facial motoneurons (69, 70), supporting our neuroanatomical data. Moreover, this area is important for the blink reflex using both electrophysiological (69) and neuroanatomical techniques (71). We conclude the retrogradely labeled neurons near the Vi/Vc junction are lamina V neurons, similar to those found more caudally. There is extensive evidence that identified lamina V neurons as important in pain pathways (72–74). These neurons usually show wide dynamic range mechanoreceptive sensitivity over large receptive fields, similar to many of the cells in the Vi/Vc transition zone (41, 43). Both lamina V neurons and those in the Vi/Vc transition zone also project to the contralateral thalamus and other places considered part of the trigeminothalamic tract. We propose that many lamina V neurons also are integral interneurons in reflex pathways. Their input from multiple fiber types, large size with dendrites extending through the dorsal horn into lamina II (75–77) and projections to somatic motor nuclei, support this view.

Descriptions of simple reflex circuits are rare, but there are examples in the spinal cord. Lamina V neurons have been confirmed electrophysiologically as premotor neurons (78–81), making them potential interneurons in reflex circuits. In this regard, seminal communications from the Schouenborg laboratory (46, 82) have shown neurons in lamina V are important interneurons in the nociceptive withdrawal reflex, a well-defined sensorimotor action where receptive field location and sensitivity distribution closely mirror the efficacy of skin withdrawal of the output muscle (83). Our data compare favorably with this model—somatotopically appropriate lamina V neurons in the trigeminocervical complex project to somatotopically appropriate groups of facial motoneurons, despite a degree of convergence in lamina V of primary afferent projections from the head and neck. We must remind ourselves however that the rostral MDH receives many sensory fibers from peripheral areas covered by mucosae, which have few projections into laminae III–IV, suggesting that somatotopy is registered best in lamina II. The transfer of afferent input to neurons in the deep dorsal horn is either directly by sensory fibers or indirectly *via* interneurons in more superficial laminae; in either case, such transfer must be substantial. It also implies the dorsoventral distribution of the dendritic trees of lamina V neurons cannot predict accurately the response profiles of their receptive fields. Thus, glabrous surfaces, such as mucosae, must direct appropriate reflex activity through lamina II. While we show herein lamina V interneurons project to appropriate somatic motor neurons in the facial motor nucleus, a previous study (12) showed numerous neurons in lamina V also were retrogradely labeled after injections of FG into rostral and caudal ventrolateral reticular formation. These injections included somatic motoneurons of the nucleus ambiguus, which innervate numerous striated muscles of the pharynx and larynx. Thus, lamina V neurons may be important for similar disynaptic reflex pathways to these neck muscles.

While there were no trigeminal neurons in lamina II retrogradely labeled after our facial injections, numerous neurons in lamina II were labeled in the rostral MDH near the Vi/Vc junctional area after injections into the nucleus tractus solitarii, as well as after injections into the rostral and caudal ventrolateral reticular formation (12). This was surprising since lamina II neurons are usually considered local interneurons. Such projections are seldom described—the very small size of lamina II neurons makes their nuclear/cytoplasmic ratio close to unity. Thus, the cytoplasmic labeling of a retrograde marker is very difficult to discern in the minimal cytoplasm present. Nevertheless, intracellular injections of neurons in lamina II show that many do indeed project out of the MDH with many having axons ascending to the reticular formation (84). We suggest neurons such as these were retrogradely labeled after injections into these reticular areas, all important for visceral function, and suggests that such neurons in lamina II near the Vi/Vc junction may be important interneurons for modulating somatovisceral reflex behavior.

The present discussion of trigeminal reflex behavior focused on the trigeminocervical complex and emphasized projections from lamina V neurons to the motoneurons innervating striated muscles in the head and neck. We also suggest connections to somatovisceral reflex pathways arise from lamina II interneurons. It is of interest that neurons in the subnucleus oralis of the spinal trigeminal nucleus are morphologically similar to neurons in lamina V of the trigeminocervical complex. These neurons receive dense projections from intraoral structures, much of which is nociceptive, and send numerous projections directly to the trigeminal motor nucleus, where motoneurons innervating the striated muscles of mastication lie (58, 85–90). Dorsomedial neurons in the subnucleus oralis are considered important as premotor to the trigeminal motor nucleus for jaw reflexes; we consider them as closely associated with lamina V neurons found more caudally and as interneurons in reflex behavior.

## Summary and Perspectives

Although “dermatomes” by definition do not exist in the MDH, our data support the hypothesis in humans (8) of sequential bands of innervation continuing from rostral cervical dermatomes over the facial skin and then going intraorally (Figure 5), and finally transitioning to visceral structures in the throat *via* the paratrigeminal nucleus. Such a configuration of “cranial dermatomes” solidifies continuity of a pattern seen in the body represented in the spinal dorsal horn as the classic dermatomes. Our tract-tracing studies show the somatotopic map of the trigeminocervical complex is reinforced by topographic projections to the facial motor nucleus. These projections suggest that orofacial receptive fields help direct functional behaviors such as eating, blinking, vibrissae whisking and ear movement. Since nearly all such projections are from lamina V of the dorsal horns, it promotes these neurons as vital links in orofacial reflex circuitry and implicates them in potential disynaptic reflexes.

**Figure 5:** Schematic of a rat’s face showing concentric lines arbitrarily drawn similar to those drawn in the human summarizing an “onion skin” hypothesis of facial innervation. The bands of color are transposed from Figure 1 and impose the central representation of nerves in the trigeminocervical complex innervating oral and perioral receptive fields (shaded red) in the rostral medullary dorsal horn (MDH) followed successively by nerves innervating the snout (shaded green), periocular (shaded blue), and periauricular (shaded orange) areas in more caudal areas of the trigeminocervical complex. This illustration thus mimics the existence of hypothetical “cranial dermatomes” and supports their continuity with spinal dermatomes for central orofacial representation.

Body images are seldom, if ever, shown over either the medullary or spinal dorsal horns. Somatotopy in spinal dorsal horns is especially difficult to picture since the relatively large nerves innervating the limbs have wide receptive fields, represented centrally over several segments of the spinal cord. Receptive fields of trigeminal nerves are relatively small and thus have a more localized central representation. Moreover, several regions in the head and neck are unique receptive fields (e.g., cornea, conjunctiva, whiskers, oral and nasal mucosa, teeth), each eliciting a different reflex when stimulated. Unlike the long columns of motor neurons innervating various limb muscles that are intermixed in the spinal ventral horn, facial motor neurons are arranged in a musculotopy, with the muscles surrounding eyes and ears found dorsally while those of the snout and nares found most laterally.

This organization is ideal for study of reflexes of the head and neck, but also studying reflexes in general. The generally small size of the spinal cord hinders experimental approaches to studying reflexes of the limbs, but the spatial separation of at least several millimeters of sensory fibers and associated interneurons from facial motoneurons promotes the study of numerous facial reflexes. While many orofacial behaviors use complex circuits with several interneurons, we believe there are also numerous simple reflexes, using only three to four neurons that direct many simple behaviors. The data offered herein may provide a substrate for studies on such behaviors. These data also provide a perspective for the neurologist to consider when diagnosing perturbations of somatosensation in the head and neck of afflicted patients.

## Ethics Statement

All protocols were approved by the Animal Care Committee of Saint Louis University and followed the guidelines published in the Guide for the Care and Use of Laboratory Animals.

## Author Contributions

WMP performed the experiments, analyzed the data, helped prepare the figures, and wrote the manuscript. BP analyzed the data, and helped prepare the figures, and assembled the manuscript. QG helped perform the experiments, processed tissues, and helped analyze the data.

## Conflict of Interest Statement

The authors declare that the research was conducted in the absence of any commercial or financial relationships that could be construed as a potential conflict of interest.
